# Effect of platelet-rich plasma on the healing of cutaneous defects exposed to acute to chronic wounds: a clinico-histopathologic study in rabbits

**DOI:** 10.1186/s13000-015-0327-8

**Published:** 2015-07-02

**Authors:** Omid Ostvar, Sahar Shadvar, Emad Yahaghi, Kamran Azma, Amir Farshid Fayyaz, Koorosh Ahmadi, Iradj Nowrouzian

**Affiliations:** Department of Pathology, Faculty of Veterinary Medicine, University of Tehran, Tehran, Iran; Brain and Spinal Injury Research Center, Tehran University of Medical Sciences, Tehran, Iran; Baqiyatallah University of Medical Sciences, Tehran, Iran; Department of Physical Medicine and Rehabilitation, Clinical Biomechanical and Rehabilitation Engineering research center, AJA University of Medical Sciences, Tehran, Iran; Department of Legal Medicine, AJA University of Medical Sciences, Tehran, Iran; Department of Emergency Medicine, Alborz University of Medical Science, Karaj, Iran; Department of Clinical Sciences, Faculty of Veterinary Medicine, University of Tehran, P.O. Box 14155–6453, Tehran, Iran

**Keywords:** Platelet-rich plasma, Histopathology, Wound, Regeneration, Rabbit

## Abstract

**Background:**

Platelet-rich plasma (PRP) contains numerous growth factors to promote wound healing and angiogenesis. The aim of this study was to gain further information about the benefits of platelet-rich-plasma for healing cutaneous acute to chronic wounds.

**Methods:**

A total of 30 New Zealand albino rabbits (*n* = 15/group) were randomly assigned to two experimental groups: control group, and PRP group. Bilateral resection defects measuring 3 cm were surgically created on the dorsolateral of the cutaneous in animals and the defects were randomly divided into two mentioned groups. Wound area, neovascularization, size and epithelialization were compared on days 7, 14 and 21 post-wounding. Histopathological analyses were conducted on 15 specimens from each group after sacrifice by the cellular aspects of the regeneration of the tissue.

**Results:**

Our results were indicated that the wound area of PRP was smaller than that in the non-treated group on days 7, 14 and 21. Furthermore, a *significant decrease of the wound size* was observed in PRP groups that were *significantly greater than that in the control group.* A significant increase of the mean vascular density was noted in the PRP treated groups compared to the control groups at day 14 and especially day 21. This results indicated that PRP treated group’ enhanced angiogenesis at the wound beds as compared to no treatment group.

**Conclusion:**

These results could be useful for researchers in the growing fields of tissue repair and experimental wound healing. Further studies will be essential to determine the role of PRP in clinical practice.

## Background

Platelets play a central role in hemostasis and wound healing. The latter is mediated by release of secretory proteins on platelet activation, which directly or indirectly influences virtually all aspects of the wound healing cascade. A recent strategy to promote the wound-repair cascade is to prepare an autologous platelet concentrate suspended in plasma, also known as platelet-rich plasma (PRP), that contains growth factors and administer it to wound sites [1, 2].

Wound regeneration commonly begins with clot formation and platelet degranulation, leading to the release of multifarious cytokines and coagulation factors, which modulate inflammatory response. To date, more than 30 various cytokines have been detected in platelets. Among those, platelet derived growth factors (PDGFs), transforming growth factors (TGFs), vascular endothelial growth factor (VEGF)*,epidermal growth factor* (EGF), and Insulin-like growth factor (IGF) has been described that stimulate cellular migration, proliferation and angiogenesis for successful wound healing [3]. Platelet gel is produced by mixing two solutions: PRP and calcified thrombin solution. The PRP can be prepared by aphaeresis or can be separated from fresh anti-coagulated blood by simple centrifugation, which concentrates platelets up to six times the baseline count in whole blood [4]. Animal studies and human trials revealed successful results in regenerative potential of PRP, suggesting that the administration of growth factors may be combined with tissue regeneration techniques in the repair of intra-bony defects, furcation’s, and cyst cavities to improve the outcome of these treatments [5–9].

Furthermore, PRP was used in the treatment of chronic cutaneous and soft tissue ulcerations [10–12]. There have been numerous publications on the use of PRP for clinical applications in periodontal and oral surgery [8, 11–14], maxillofacial surgery [10–13], orthopedic and trauma surgery [14–18], cosmetic and plastic surgery [19, 20], spinal surgery [10, 11], heart bypass surgery [10], and burns [21]. Platelets in PRP also play a role in host defense mechanism at the wound site by producing signaling proteins that attract macrophages [13]; PRP also may contain a small number of leukocytes [17, 20] that synthesize interleukins as part of a non-specific immune response.

## Methods

### Ethics statement and animals

All experimental protocols were approved by the local animal care committee in accordance with Faculty of Shiraz Veterinary Medicine office regulations. In current study, 30 New Zealand albino rabbits of both sexes, weighing 2400–4700 g, with averagely 3 weeks old were selected. The animals were kept two by two in individual propylene cages under standard laboratory conditions by the dimensions of 45 × 60 × 90 cm^3^. Rabbits were maintained on a 12 h light/dark cycle at 22 ± 1 °C and 50 ± 10 % humidity, and fed with standard rat diet and water ad libitum.

#### PRP preparation

Rabbit blood was collected from healthy animals in an EDTA-coated container (BD Vacutainer®, Franklin Lakes, NJ). PRP was isolated as previously described [21]. The blood was centrifuged at 2,400 rpm for 10 min at room temperature. After discarding the upper platelet-poor plasma, the sample was further centrifuged at 3,500 rpm for an additional 15 min, thereby separating the upper PRP layer and the lower red blood cells- and white blood cells-rich layer. The upper layer was collected carefully using an auto-pipette.

### Wound treatment

A rabbit model of hemorrhagic shock was established as described previously. Briefly, New Zealand albino rabbits were anesthetized via intramuscular injection of ketamine (21 mg/kg body weight) and xylazine (2.2 mg/kg body weight). A 3 cm sized skin defect was created on the back of each rabbit with surgical scissors. Epidermis, dermis, and SC were removed, and the muscle fascia was exposed. In order to prevent the wound by contracture, 4 sutures were placed at the border of the wound with 6–0 sutures (Ethicon, Somerville, NJ) and the wound margins were anchored to the underlying muscle fascia. The wounds were treated once with a total 200 μl of PRP (*n* = 7). PRP was formed on the wounds by directly applying 100 μl of PRP on each of the wounds and the wounds were covered with polyurethane film. The films covering the wounds were changed every 7 days to take macroscopic pictures of the wounds. Platelet-rich plasma (PRP) was separated by centrifugation for 15 min at 300 xg, and the plasma proteins were concentrated together with the platelets using the cold ethanol precipitation method. The animals were individually housed after surgery. The animal study procedures were approved by the Institutional Animal Care and Use Committee at Shiraz University.

### Experimental protocol and evaluation of wound healing

The rabbits *were randomly allocated* into two groups, each group containing fifteen submitted animals. Two symmetrical wounds were created on either side of the back of each rabbit that were made in the laterodorsal cutaneous. It is worth noting that one wound was as control group and *PRP* was *applied* on *wound* in *PRP group* (Fig. 1). Both wounds were then covered with a polyurethane film, and evaluated macroscopically and histologically on days 7, 14 and 21 after the operation.

**Fig 1:** Cutaneous lesions of PRP rabbit after 1 week: the lesion is humid and non to mild -exudative, with marginal epithelization starting from the lesion edges, the wound is <100 % epithelialized, with marked fibrin deposition. There is moderate erythema of the peri and intra-wound area and firm

The wounds were evaluated macroscopically and histologically. For macroscopic evaluation of wound healing, each wound edge was traced and all rabbits were euthanized of the surgical procedure by *carbon dioxide inhalation* at days 7, 14 and 21. The wounds were sampled in full-thickness, including the underlying muscle. For the biopsy, we used an 8-mm diameter dermal biopsy punch (Stiefel Laboratories®). All specimens were used for histological analysis. The histological specimens were fixed in formalin, embedded in paraffin, sectioned transversely (4 μm tick). Then, *transverse sections were* stained with hematoxylin and eosin *(H&E*) *for histological examination*.

## Results

### Observation and closure of macroscopic wounds

The wounds were evaluated macroscopically and histologically on the 7th, 14th and 21st after the wound creation. Totally, the macroscopic findings in the PRP-treated groups were improved and organized than the control groups (Figs. 1, 2 and 3). On the other hand, the percentage decrease of the wound size in PRP groups was significantly greater than that in the control group, which these findings showed a significant difference in the percentage decrease of the wound area between the PRP and control groups (Figs. 1, 2 and 3). The PRP group was demonstrated significantly smaller wound size compared to the non-treated groups at days 14 and 21. The wound sizes of control groups were not significantly different from those of no treatment group at day 14 and day 21.

**Fig 2:** Wound area on day 14. Percentage decrease in the wound size. The generation of granulation tissue and the re-epithelialisation observed in the wounds covered with PRP are clearly superior to that in the control wound, which shows few signs of healing; there is mild erythema of the peri-wound area and firm, black granulation tissue in the wound bed

**Fig 3:** Day 21 of cutaneous wound healing with PRP in the treatment group: The wound has healed after tree applications of PRP; the wound is clearly contracted in all dimensions. The margins are intact, and there is noticeably less bleeding with debridement. And also, the percentage decrease in the wound size was significantly greater in the week 3 as compared with 14 days expressed

### Histological observation

The histopathological examination indicated that there were significant *differences* in the pattern of *wound healing* among the two groups. There were significant differences between the treated groups with PRP and control group in the mean percentage of collagen fibres at days 14 and 21. Furthermore, by day 7, there were increased newly organized collagen bundles and relatively advanced epithelium at the wound junction of PRP-treated wounds revealed as compared to non-treated wounds (Fig. 4). In parallel, on day 7, several small vessels (angiogenesis) were also apparent in the PRP treated tissues, whereas only a few vessels were present in control tissues. Because organized collagen fibers give tensile strength to the tissue, the arrangement of collagen observed in the experimental group is consistent with tissues that possess good tensile strength and improved wound healing. A significant increase of the mean vascular density was noticeable in the PRP treated groups compared to control groups at day 14 and especially day 21. Therefore, it can be concluded that PRP treated group’ enhanced angiogenesis at the wound beds in comparison with no treatment groups (Figs. 5 and 6). Moreover, by days 14 and 21, all wounds contained abundant fibroblasts and collagen bundles, through rich neovascularization were detected only in the PRP-treated wounds (Figs. 5 and 6). Furthermore, in PRP group, inflammatory responses were observed at *lower frequency* range than the control groups at 14 and 21 days. It is worth noting that the results were better in study group than in the control group**.**

**Fig 4:** Post-wound tissue stained with hematoxylin and eosin. Representative skin from a PRP wound 7 days after wounding with increased inflammatory cells and new collagen fiber bundles are sparse, which these fibers do not fill in between the intact collagen bundles (200Ҳ, B = 10 μm)

**Fig 5:** Histopathologic section of wound related to treatment group, 14 day post-wounding, indicates vascular density on day14. Tissue from the PRP-treated wound at day 14. New collagen bundles filled densely, new blood vessels are found in the deep dermal layer only in the PRP-treated wounds (H&E,200 Ҳ B = 10 μm)

**Fig 6:** Photomicrograph in experimental all groups in cutanenous wound at 21th day. Mature epithelial cells are obvious in PRP treated wounds obtained 21 days after wounding. Proliferative activity in the epidermis is higher in this tissue, Note complete wound healing. The presence of epidermis layer cover the mature granulation tissue (H&E,400 Ҳ B = 20 μm)

## Discussion

Emerging new therapies such as PRP can have an adjunctive role in a standardized, quality treatment plan. The application of autologous PRP to soft tissue healing has been a subject of great interest for much of the past two decades. Multiple growth factors are present in high concentrations within PRP. Some of the most important of these include PDGF, TGF-β, VEGF, EGF, and IGF. PDGF, TGF-β, VEGF, and EGF have been shown to be increased 3 to 7 times in autologous PRP [22, 23]. Moreover, platelet concentrates contain many powerful mitogenic and chemotactic growth factors, which regulate key processes involved in tissue repair, including cell proliferation, chemotaxis, migration, cellular differentiation, and extracellular matrix synthesis [24, 25].

The results of this study appear to confirm observations from the basic science of wound repair; in the large number of wounds, a positive change in wound variables was seen following application of physiologically relevant concentration of platelets. These findings are important because, while the PRP injection remain the gold standard for determining treatment efficacy [26]. Furthermore, we have revealed the benefits of topical platelet-rich plasma gel for the treatment of the laterodorsal cutaneous wounds. Our study have shown that wounds treated with PRP exhibited faster healing rates and adequate granulation tissue formation when compared to wounds treated with non-treated group. In addition, topical use of PRP has been shown to enhance angiogenesis in the early stage of the repair process after open skin and subsequently to promote wound healing.

According to the scope of the present study the effect of PRP in wound healing indicated similar positive result of PRP in acceleration of epithelial migration, the angiogenic response and tissue fill. In parallel, several clinical studies, in both human and veterinary medicine, on the restoration of tissue integrity have shown the positive role of platelets in natural wound healing [27–29]. When locally applied, platelets accelerate healing of normal tissue and promote healing of impaired wounds [30, 31]. Furthermore, Sharma and Maffulli have been reported that collagen is produced by epitenon cells at the initial stage of the healing process, whereas endotenon cells synthesized collagen later [32]. However, these results is in agreement with those studies induced by Lee et al., that have noted acceleration of epithelialization in treatment of lower equine wound with PRP [33] and faster resolution in inflammatory response. Moreover, Vaterio et al., have been shown acceleration in skin reepithelialization by using PRP during fat grafting in patient who underwent plastic surgery [34]. In previous study, Alsabaawe, Hom et al., have been suggested an increased of epithelialization rate and regression of acute inflammatory process in PRP treated skin wounds in rabbits during week 1 postoperative period compared to week 2 where there was no statistical differences found in epithelial thickness and inflammation stage between PRP treated wound and control. Also, they indicated that the epithelialization returned to normal texture and improvement of wound healing in term of reducing the inflammatory process [35, 36]. On the other hand, Ahmad et al., (2012) suggested that the PRP has the potential to enhance the healing of tissue at the cellular level via the recruitment proliferation, and differentiation of cells involved in tissue regeneration [37] Moreover, Gotterbarm et al., (2006) have been reported the PRP acts as a rich source of autologous growth factors [38]. Sun et al., (2010) have been mentioned that, PRP is a very good clinical source for osteochondral regeneration [39]. On the other hand, Shin et al., (2012) proved that PRP was effective in normal tissue regeneration [40]. These researches are in agreement with our study. Moreover, recent studies demonstrated that histopathological examinations are gold standards as diagnostic criteria in the experimental animals on the different fields [41–45].

## Conclusions

The results of systematic review and hisological analysis revealed that wound healing time of PRP treatment group was shorter than that of control group. These results could be useful for researchers in the growing fields of tissue repair and experimental wound healing. Further studies will be essential to determine the role of PRP in clinical practice. Controlled studies with sufficient sample sizes are needed to prove the efficacy of platelet-rich plasma to treat wounds.
